# Strategies of Ice and Snow Tourism to Optimize Ecological Environment and Economic Growth from the Perspective of Sustainable Development

This article has been retracted.

**DOI:** 10.1155/2022/9577859

**Published:** 2022-10-04

**Authors:** Xiejun Cheng, Donghui Zhang

**Affiliations:** ^1^School of Business, Jiangsu Second Normal University, Nanjing, 211200 Jiangsu, China; ^2^Department of Physical Education, Jinling Institute of Technology, Nanjing, 211169 Jiangsu, China

## Abstract

Due to the successful holding of the Winter Olympics, China's enthusiasm for ice and snow sports has soared, and its enthusiasm for ice and snow tourism has also been further stimulated. At present, most of China's ice and snow tourism (IST) attractions are concentrated in the three eastern provinces. At the same time, due to the increasingly harsh environment, the natural landscape of IST is also shrinking. Therefore, this paper aims at studying the strategies of IST to optimize the ecological environment and economic growth from the perspective of sustainable development. First of all, this paper makes a certain introduction to the current situation of IST. After that, the current IST resources in China were analyzed, and the three northeastern provinces were taken as the research objects, and the distribution location, traffic conditions, and development trends of IST resources were studied in detail. Then, the autoregressive model is used to fit the tourism resources and tourist growth with the economic growth, and combined with the trend shown by the economic growth model, a strategy for the sustainable development of IST is proposed. The experimental results of this paper prove that the regional system attribute of IST resources and economic growth model is between 3 and 5, and the average is about 3.6, which shows that the growth of tourism resources has a positive correlation with economic growth. Therefore, from the perspective of sustainable development, the economic growth of the IST industry should also focus on the protection and humidity development of natural ice and snow landscapes.

## 1. Introduction

Due to the early development time, North America and Europe have become the first regions in the world to develop IST. This has brought a series of influences, including a general consensus among people in the world. After turning the field of vision to the country, it is found that the development characteristics of the domestic IST industry are somewhat different from those of foreign countries. The three northeastern provinces with Heilongjiang as the core in China are the regions that developed ice and snow tourism earlier. With the passage of time, in the past 50 years, North China, Northwest China, and Southwest China have also begun to develop ice and snow tourism, and gradually formed a trend. China's winter ice and snow tourism industry is on the right track, and the ice and snow tourism market continues to heat up. In recent years, the improvement of material conditions has made people's awareness of sports continue to increase. Sports awareness is the forerunner of healthy life, and the people's enthusiasm for participating in sports activities is getting higher and higher. When there is demand, there will be supply, and various festivals based on sports activities have begun to enter people's lives. Taking ice and snow sports as an example, the ice and snow festivals based on ice and snow sports in various places have developed with the growth of people's sports awareness and enthusiasm. The holding of these ice and snow festivals has become a business card for local cities. They play a role in stimulating economic development, enriching urban culture, promoting the popularization of related ice and snow sports, improving people's physical fitness, and enriching people's spiritual and cultural life. Therefore, based on the perspective of sustainable development, it is necessary to study the strategies of IST to optimize the ecological environment and economic growth.

IST has always been a tourism project that people yearn for and have been trying, and the proportion of IST in the tourism economy is on the rise. In this regard, more and more scholars have studied the economy and industry of IST. Wen studied the economy of the IST industry based on the perspective of the Olympic Games. He used the enthusiasm for ice and snow sports brought by the Winter Olympics as a variable to establish a model that IST promotes the growth of the ecological environment [1]. Taking 832 impoverished counties in China as a sample, Hong-Min et al. proposed the Integrity Suitability Index (ISI) based on natural and socioeconomic factors to evaluate the suitability and potential of IST in impoverished counties [2]. Ziegler et al. aimed to explore whether ecotourism work alters local people's perceptions, attitudes, and behaviors toward key species and their habitats, and if so, whether the type of tourism influences these outcomes [3]. Falk and Vieru studied the local climate; that is, the time and amount of snowfall in winter and the influence of tourists' overnight accommodation. His research data model shows that the impact of natural snow conditions on overnight stays varies by country of origin [4]. Li et al. took the integrated development of the ice and snow industry and the health industry in Tieli and Genhe as examples. The necessity and basic conditions for the integrated development of the ice and snow industry and the health industry were discussed, and the “ice and snow+health” product system was initially designed [5]. However, their analysis of the IST market is more of a macroanalysis from the policy aspect and lack of specific analysis of specific regions.

The ice and snow economy is also an economy based on natural ice and snow landscapes. How to achieve sustainable development based on ecological environmental protection is also a problem that many scholars study. Liu developed a new sustainability index that emphasizes environmental justice to better classify and assess ecocities [6]. ZiYi et al. proposed the Ecological-Living-Productive Land (ELPL) classification system, which aims at guiding China's land pattern to take an ecologically centered path, and the development model will shift from a single function to a more comprehensive multifunctional land use [7]. Thiers et al., taking the Portland metropolitan area as an example, studied the trend of the ecological environment under urban development and studied the role of state government policies in shaping and supporting different institutions [8]. Based on the principle of minimizing environmental and ecological impacts, Chen established an ecological economic system model to conduct research on China's industries [9]. However, their research did not make an in-depth discussion of the key word of ice and snow economy but only studied the coupling relationship between the environment and the economy in the general environment.

The innovation of it is that, according to the data of China's IST economy, tourism resources and number of tourists, through the long-term tracking of the study area, people can grasp the internal connection between economic growth and the natural ecological environment. China's IST economy is constantly developing, and the economy of IST is also changing. With the rapid growth of the IST market economy, various contradictions between the traditional growth mode and the ecological environment are intertwined. To achieve the coordinated development of sustained economic growth and natural ecological environment will inevitably become the top priority for China's economic development for a long time in the future. In addition, while conducting theoretical and methodological research, it pays more attention to serving the practical needs of sustainable economic development.

## 2. Sustainable Development of IST Industry

### 2.1. IST Industry

Based on the natural environment, ecological environment and cultural environment of ice and snow are needed to have a deep understanding of the meaning and research objects of ice and snow culture. According to the literature review and its characteristics, the specific definition of ice and snow culture is summarized:

The production of ice and snow culture originates from the natural and human environment. People use ice and snow as the basic elements to transform the ice and snow ecological environment, resulting in a life formed with ice and snow connotations, as shown in Figure 1 [10].

In recent years, the three northeastern provinces have been striving to build IST brands, making use of the region's unique, natural, and geographical advantages to vigorously develop IST. Heilongjiang takes the “Crown of Ice and Snow, Cool Longjiang” as its brand to promote the creation of IST themed products, involving a number of tourism industries including ice and snow sports, landscape, hunting, hot springs, and study tours. As shown in Figure 2, it is a variety of IST projects [11].

In the winter of 2018-2019, more than 20 million tourists from outside the province were received and the number of tourists received by the ice and snow tourist attractions also increased by a considerable amount. Taking Harbin Ice and Snow World as an example, the year-on-year increase has reached 17.00%. Jilin Province has actively held ice and snow summits, food festivals, developed ice and snow sports, opened cross-regional ice and snow trains, and a series of ice and snow policies to innovatively solve the problems of IST [12]. In the 2017-2018 snow season, the province received 72.6389 million tourists, a year-on-year increase of 17.18%, and realized ice and snow tourism revenue of 142.181 billion yuan, a year-on-year increase of 22.57%, accounting for 36.85% of the province's average total tourism revenue. During the Spring Festival of 2018 alone, Liaoning Province received 20.32 million tourists, and the tourism revenue reached 14.5 billion yuan. Many large ski resorts received an average of nearly 2,000 tourists per day, a significant increase over the same period last year. As shown in Figure 3, for the famous Harbin Ice Sculpture, there are many tourists who go to Harbin for the Ice Sculpture Festival every year.

### 2.2. Ecological Sustainable Development

In the context of rapid global population growth, increasingly scarce resource management and further deterioration of the ecological environment, the theory of sustainable development emerged. The “Our Common Future” report is the first to put forward the theory of sustainable development and define sustainable development as development that meets current development needs without jeopardizing the ability of future generations to meet their needs. Sustainable development involves economy, resources, environment, population, etc. and follows the principles of fairness, continuity, and commonality. From the perspective of marine economic geography, the sustainable development of the marine economy emphasizes the importance of the relationship between people and the sea. By coordinating the relationship between man and sea, economy and environment, and contemporary and future we can realize the coordinated and balanced development between man and sea and society [13]. In the field of marine research, the basic idea of sustainable development mainly includes three aspects: First, pay attention to marine resources and quality. The growth of the marine economy should take into account the coordinated development of quality and quantity and change the growth mode of the marine economy. That is, relying on scientific and technological innovation and progress, improving the quality of production management elements and labor productivity to expand the scale of production and operation for analysis and transformation. Secondly, natural resources and environmental carrying capacity are the basis for the development of marine economy; third, it emphasizes the comprehensive and healthy development of human society [14].

### 2.3. Vector Autoregression (VAR) Model

Vector autoregression model (VAR) is a commonly used econometric model, which is widely used to explore the dynamic relationship between variables. The two-dimensional p-order VAR linear model constructed in this paper is as follows [15]:

(1) $$\begin{array}{c} Z_{t}=v+z_{t-1}\cdot \delta_{1}+\cdots +z_{t-q}\cdot \delta_{p}+\beta_{t}. \end{array}$$

In the formula:

(2) $$\begin{array}{c} z_{t}={\left(y_{1t},y_{2t}\right)}^{\prime }. \end{array}$$

In the formula, *z*_1_ is the IST resource variable, *z*_2_ is the economic variable, *δ*_1_, ⋯, *δ*_*p*_ is the regression coefficient, and *β*_t_ is the error term.

When the regression coefficient and mean value of the main error distribution in Formula (1) are assumed to be constant constants, the autoregressive model's description of the relationship between economic growth and IST resources exhibits the properties of time series stationarity. However, the structure of the model adjusts if the time series' structure changes abruptly at various points. The latent nonlinear properties of the time series of endogenous variables cannot be reliably shown by Formula (1), which can only express the linear connection [16]. Therefore, in order to accurately describe the internal relationship between economic growth and ice and snow tourism resources, this paper introduces a nonlinear “regional system transfer” factor and assumes that the parameters of the model change with the regional system transfer of the economic system. Markov's zoning transition model is as follows:

(3) $$\begin{array}{c} Z_{t}=\mu \left(S_{t}\right)+\overset{q}{\underset{i=1}{\sum }}\varphi_{i}\left(S_{t}\right)z_{t-q}+\varepsilon_{t},\\ \varepsilon_{t}\left|I_{t-1}\sim iidN\left(0,\sigma_{S_{t}}^{2}\right)\right.. \end{array}$$

In an MS-VAR model, the Markov chain generates *S*_*t*_ as follows:

(4) $$\begin{array}{c} p_{r}\left[S_{t}\left|{\left\{S_{t-1}\right\}}_{i=1}^{\infty }\right.,{\left\{Z_{t-1}\right\}}_{i=1}^{\infty }\right]=p_{r}\left\{S_{t}\left|S_{t-1};\rho \right.\right\}. \end{array}$$

Among them, it is assumed that *S*_*t*_ has m zoning states; that is, *S*_*t*_ ∈ {1, 2, ⋯, *m*} and *ρ* contain probability parameters. Definition *p*_*ij*_ the transition probability from state *i* at time *t* − 1 to state *j* at time *t* − 2, namely

(5) $$\begin{array}{c} p_{ij}=p_{r}\left(S_{t}=j\left|S_{t-1}=i\right.\right),0<p_{ij}<1,\\ \overset{m}{\underset{j=1}{\sum }}p_{ij}=1. \end{array}$$

Therefore, the transition probability matrix of *p*_*ij*_ has the following form:

(6) $$\begin{array}{c} p_{ij}=\left[\begin{array}{cccc} p_{11} & p_{12} & \cdots & p_{1m}\\ p_{21} & p_{22} & \cdots & p_{2m}\\ \vdots & \vdots & \cdots & \vdots \\ p_{m1} & p_{m2} & \cdots & p_{mm} \end{array}\right]. \end{array}$$

According to the AIC and SC information criteria, the MS-VAR model [17, 18] containing two regional systems is adopted, namely

(7) $$\begin{array}{c} Z_{t}=\left[\begin{array}{c} Z_{1t}\\ Z_{2t} \end{array}\right],\\ Z_{t}=\left[\begin{array}{c} \mu_{1},S_{t}\\ \mu_{2},S_{t} \end{array}\right]+\overset{q}{\underset{i=1}{\sum }}\left[\begin{array}{cc} \varphi_{11},s_{t} & \varphi_{12},s_{t}\\ \varphi_{21},s_{t} & \varphi_{22},s_{t} \end{array}\right]\left[\begin{array}{c} Z_{1t-q}\\ Z_{2t-q} \end{array}\right]+\left[\begin{array}{c} \varepsilon_{t}\\ \omega_{t} \end{array}\right]. \end{array}$$

Among them, *z*_1*t*_ represents the variable of IST resources and *z*_2*t*_ represents the economic variable, namely

(8) $$\begin{array}{c} z_{t}={\left({\text{solid}}_{t},{\text{eco}}_{t}\right)}^{\prime },\\ z_{t}={\left({\text{liquid}}_{t},{\text{eco}}_{t}\right)}^{\prime }. \end{array}$$

Among them, solid_*t*_ represents the time series of the growth rate of the ice and snow resources, while liquid_*t*_ represents the time series of the growth rate of the tourism industry using the ice and snow resources. The name for random disruption is *ε*_*t*_, *ω*_*t*_, assuming that the state-dependent nature of the model's parameters and their dependence on the *S*_*t*_ zoning state variable. The model's zone state variable transition probability matrix has the following shape since the transition probability between the two zones simultaneously fulfills the first-order Markov chain:

(9) $$\begin{array}{c} p=\left[\begin{array}{cc} p_{11} & p_{12}\\ p_{21} & p_{22} \end{array}\right]. \end{array}$$

The Expectation Maximum (EM) algorithm is an optimization algorithm based on the Maximum Likelihood Estimation (MLE) theory.

## 3. IST Resources in the Three Northeast Provinces

As of April 2019, the statistics of the number of IST resources in the three northeastern provinces are shown in Figure 4. The darker the color, the more abundant the tourism resources are. The interprovincial distribution of IST resources in the three northeastern provinces is quite different. Heilongjiang and Liaoning have the same number, accounting for nearly 40%, and Jilin Province has only half of the other two provinces [19]. Comparing the number of ice and snow tourism resources in each province with the average of the three provinces, Jilin Province is far below the average, while Heilongjiang and Liaoning provinces are both above the average, but the difference in quantity is not obvious.

According to the five categories of sports, ice and snow recreation, folk festivals, landscape viewing, and hot spring recuperation, the types of IST resources in the three northeastern provinces are classified and counted, as shown in Figure 5. The types of IST resources in the three northeastern provinces are dominated by sports, accounting for about 34.2% of the total; landscape viewing and folk festivals are less, accounting for 10.5% and 8.9% of the total, respectively. The number of ice and snow amusement and hot spring recuperation is in the middle, accounting for about 46.4% of the total.

The tourism scale index can show the specific situation of the quantity and quality of the ice and snow tourism resource scenic spots in each region from a macroperspective, which is of great value for understanding the development and evolution of the research site. The scale index is the ratio of the number of regional scenic spots to the regional area [20]. The calculation formula is as follows:

(10) $$\begin{array}{c} G_{i}=\frac{n_{i}}{A_{i}}. \end{array}$$

*G*_*i*_ is the scale index; *i* is the *i*-th study area (prefecture-level city/province); *n*_*i*_ represents the number of IST resources in the *i*-th study area; and *A*_*i*_ represents the area of the study area. It can be seen from the formula that when the area of the study area is fixed, the scale degree index is positively correlated with *n*_*i*_. The larger the scale degree, the more relative the quantitative advantage of IST resources in this area. Calculated according to Formula (10), the scale index of IST resources in the relevant area can be obtained, and the result is shown in Figure 6.

Overall, Liaoning Province has the largest scale of IST resources, twice the scale of the three northeastern provinces. The scale of IST resources in Heilongjiang and Jilin provinces is lower than the overall scale of the three provinces and far lower than that of Liaoning Province. Comparing the scale of IST resources by type, no matter what kind of IST resources, the scale of Liaoning Province ranks first in the three eastern provinces and is significantly higher than the overall scale of the three provinces. In addition, although the overall scale of Heilongjiang Province is smaller than that of Jilin Province, the scale of ice and snow tourism resources of folk festivals and festivals is slightly higher than that of Jilin Province. According to the scale degree index, although the IST resources in Heilongjiang Province have an advantage in quantity, due to the vast territory, the scale degree has been reduced. Among the smaller Liaoning and Jilin provinces, although the number of IST resources in Liaoning Province is in the middle, it has the highest scale. Although Jilin Province has the least amount of IST resources, the scale degree has been fluctuating in a small range up and down the overall scale degree.

The nearest neighbor analysis method refers to the geographical index of the proximity of point-like objects in geographical space. It can reflect the agglomeration degree of the spatial distribution of tourism resources within a certain area and is widely used in the study of tourism spatial structure. Calculated as follows:

(11) $$\begin{array}{c} r_{E}=\frac{1}{2\sqrt{n/A}}=\frac{1}{2\sqrt{D}},\\ R=\frac{r_{i}}{r_{E}}. \end{array}$$

Kernel density can be used to analyze the spatial distribution and aggregation of IST resources in the three northeastern provinces. It is centered on a specific point, expands outward according to a specific search radius, searches for other points within the radius, and finally stops when the point density is 0. Kernel density analysis can clearly reflect the aggregation form of IST resources in a specific geographical range through intuitive graphic patterns. The calculation formula is as follows:

(12) $$\begin{array}{c} f\left(x\right)=\frac{1}{\text{nh}}\overset{n}{\underset{i=1}{\sum }}K\left(\frac{x-x_{i}}{h}\right). \end{array}$$

In order to obtain a more credible kernel density measurement bandwidth *h*, this paper uses Ripley's *K*-function and uses the multidistance spatial clustering analysis tool in ArcGIS to first conduct a statistical analysis of the spatial distribution of IST resources in the three northeastern provinces. In the calculation of the multidistance spatial clustering tool, Ripley's *K*-function is commonly transformed. The transformed calculation formula is as follows:

(13) $$\begin{array}{c} \text{L}\left(\text{d}\right)=\sqrt{\frac{A\sum_{i=1}^{N}\sum_{j=1,j\neq i}^{N}k\left(i,j\right)}{\pi N\left(N-1\right)}} \end{array}$$

In Ripley's *K*-function curve figure, Exp is the expected value curve of the randomly distributed *K* function, and Obs is the observed value curve. When the confidence level is 99%, LwConf is the lowest confidence value curve, HiConf is the highest confidence value curve, and the middle is the confidence interval. When L(d) > HiConf, it is spatial clustering; when L(d) < LwConf, it is spatially discrete. As shown in Figure 7(a), taking Ripley's *K*-function curve of IST resources in Heilongjiang Province as an example, according to the curve, it is found that the Obs curve of the observed value has been on an upward trend. The difference curve Diff between the observed value and the expected value continues to rise in the distance unit of 0-0.8. When the distance unit is greater than the interval of 0.7-0.8, it shows a clear downward trend. After careful analysis, it is found that the dividing line of the curve change is 0.74. This is consistent with the clustering and discrete changes of the L(d) function curve in the confidence interval. When the distance unit is lower than 0.74, L(d) > HiConf is spatial clustering, otherwise it is spatially discrete. Therefore, when carrying out the nuclear density analysis of Heilongjiang Province, 0.74 is used as the bandwidth value, and then the nuclear density analysis is carried out. Similarly, as shown in Figures 7(b) and 7(c), the core density bandwidth of IST resources in Jilin Province should be 0.27, that in Liaoning Province should be 0.35, and the overall core density bandwidth of the three northeastern provinces should be 0.94.

In order to further understand the location of the spatial distribution of IST resources in the three northeastern provinces, the standard deviation ellipse model was used. The standard deviation ellipse takes the average center of each data point in the study area as the starting point and calculates the standard deviation of the abscissa and ordinate coordinates of all data points to obtain the long and short axes of the standard deviation ellipse, and then creates the ellipse of these data points. Through the standard deviation ellipse, it can be intuitively seen whether the distribution of point elements in the study area has a specific direction, which provides a certain reference value for the spatial distribution direction of IST resource points. The calculation formula is as follows:

(14) $$\begin{array}{c} {\text{SDE}}_{x}=\sqrt{\frac{\sum_{i=1}^{n}{\left(x_{i}-\bar{X}\right)}^{2}}{n}},\\ {\text{SDE}}_{y}=\sqrt{\frac{\sum_{i=1}^{n}{\left(y_{i}-\bar{Y}\right)}^{2}}{n}.} \end{array}$$

Among them, SDE_*x*_ and SDE_*y*_ are the major and minor axes of the standard deviation ellipse and *n* is the number of all points; *x*_*i*_ and *y*_*i*_ are the abscissa and ordinate of the *i* point and $\bar{X}$ and $\bar{Y}$ are the average center of all points, that is, the center of the standard deviation ellipse.

## 4. Deconstruction of Tourism Resources and Economic Growth Model

This paper uses the ADF test method to test the stationarity characteristics of the time series. The results show that the economic growth rate and the growth rate of ice and snow tourism resources are stable at the 1% significant level. And according to the AIC and SC information criteria, the nonlinear MSMH(M)-VAR(p) model with the number of zoning systems of 2 and the lag order of 1 is constructed by GUASS software.

The model of IST resources and economic growth adopts the vector autoregressive model. After input and analysis of multiple data, the MSMH(2)-VAR(1) model is determined. And the model is divided into two systems, namely the tourism resource growth and economic growth model, the solid_*t*_ − eco_*t*_system and the tourist growth and economic growth model, the liquid_*t*_ − eco_*t*_ system. Estimated results of model parameters for the three northeastern provinces are shown in Figure 8.

Figure 9(a) shows the smoothed probability values for each year when the “solid_*t*_ − eco_*t*_” system is in the “slow economic growth” and the “stage of rapid economic growth.” It can be seen that the transfer of the regional system in Heilongjiang is relatively concentrated, the transfer of the regional system in Jilin is relatively stable, and the transfer of the regional system in Liaoning is more frequent.

Heilongjiang and Jilin were in the “slow economic growth” in 2005-2009, 2010-2015, and 2018-2020, and the average smoothed probability was 1.000. Under the state of “stage of rapid economic growth”, increasing the number of IST resources and increasing the number of tourists can only unilaterally improve the ecological level of the natural environment. It will not produce a positive feedback of linkage effect on economic and social development, but will slow down the height of market economic growth.

Figure 9(b) shows the smoothed probability values for each year when the “liquid_*t*_ − eco_*t*_” system is in the “slow economic growth” and the “stage of rapid economic growth.” The transfer of the regional system in Liaoning is more frequent, and it has been in the “stage of rapid economic growth” since 2005. The transfer of the regional system in Heilongjiang is relatively concentrated, and the transfer of the regional system in Jilin is relatively stable.

The relationship between “economic growth and IST resources” in the “slow economic growth” and “stage of rapid economic growth” was further discussed in order to further explore the internal connection between the economic growth of IST and the resources. This was done on the basis of the analysis of the nonlinear periodic change law of the internal connection between China's IST economic growth and IST resources. The association coefficients between “economic growth and IST resources” in various growth zone systems are displayed in Tables 1 and 2.

By observing the correlation coefficient of the “economic growth and ice and snow tourism resources” system listed in Table 1, it is found that when the “solid_*t*_ − eco_*t*_” system is in the “low-speed growth zone system”, the growth rate of ice and snow tourism resources is negatively correlated with the economic growth rate. While in the “high-speed growth zone system”, the growth rate of ice and snow tourism resources is positively correlated with the economic growth rate.

By observing Table 2, it can be found that there is not only a “sustainable and healthy development” economic growth model between China's IST economic growth and natural ecological environmental protection but also an economic development phenomenon of “exchange pollution for growth”. Moreover, the internal connection between China's economic growth and IST resources will change with the transition of different regional systems.

Tables 3 and 4 show the results of the zoning attribute of the “Economic Growth and IST Resources” system.

Table 3 shows that with the continuous development of social economy, the IST resources of IST are in a state of continuous decline, which is consistent with the previous research results. In general, the green development model vigorously promoted by China has increased the growth of tourists, enabling IST to maintain stable economic growth while reducing environmental pollution.

From the trend analysis in Table 4, it can be seen that under the background of the continuous innovation and development of China's IST social economy, the growth rate of IST resources has accelerated. There is an economic development phenomenon of “promoting growth through pollution” among China's IST. There is a significant positive correlation between the destruction of the natural landscape of ice and snow and the mode of economic growth. On the whole, the “liquid_*t*_ − eco_*t*_” system has a high probability of being in the stage of rapid economic growth, indicating that the damage to the natural ice and snow landscape in the northeast is on the rise with economic development. Under the background of the hot development of IST, the pressure of tourists on the natural ice and snow environment has gradually become prominent, and the green development of the natural ecological environment is still facing enormous pressure.

## 5. Conclusions

From experience description to process simulation is the trend of geography development. This paper is based on the “solid_*t*_ − eco_*t*_” system composed of the growth rate of IST resources and the economic growth rate. The “liquid_*t*_ − eco_*t*_” composed of the tourist growth rate and the economic growth rate, using a two-stage nonlinear Markov zone transfer model. The analysis results of the zoning system attributes of the “economic growth and IST resources” system show that the probability of maintaining the original growth zoning system for each subsystem is greater. With the development of the economy, the number of IST resources gradually decreases, while the number of tourists increases with the development of the economy. It demonstrates that China's IST economy and natural ecological environment have a development trend in the direction of coordinated and symbiotic development in the process of economic development.

## Figures and Tables

**Figure 1:** The natural state of ice and snow.

**Figure 2:** Rich IST projects.

**Figure 3:** The world-renowned Harbin Ice Sculpture.

**Figure 4:** Distribution of tourism resources in the three northeastern provinces.

**Figure 5:** Type distribution of IST resources in the three northeastern provinces.

**Figure 6:** The scale index of IST resources.

**Figure 7:** Ripley's *K*-function curve of IST resources in the three northeastern provinces.

**Figure 8:** Estimated results of model parameters for the three northeastern provinces.

**Figure 9:** System smoothing probability.

**Table 1:** solid_*t*_ − eco_*t*_ System Intrinsic Relationship Coefficients.

solid_*t*_ − eco_*t*_	Low growth zoning		High-speed growth zone	
	solid_*t*_	eco_*t*_	solid_*t*_	eco_*t*_
solid_*t*_	1	-0.365	1	0.357
eco_*t*_	-0.3650	1	0.357	1

**Table 2:** liquid_*t*_ − eco_*t*_ System Intrinsic Relationship Coefficients.

liquid_*t*_ − eco_*t*_	Low growth zoning		High-speed growth zone	
	liquid_*t*_	eco_*t*_	liquid_*t*_	eco_*t*_
liquid_*t*_	1	0.468	1	-0.189
eco_*t*_	0.468	1	-0.189	1

**Table 3:** The zoning transition probability matrix and zoning attributes of the 2005-2020 “solid_*t*_ − eco_*t*_” system.

solid_*t*_ − eco_*t*_		Zoning transition probability matrix		Zoning attribute
		High-speed growth zone	Low growth zoning	Average duration
Heilongjiang	High-speed growth zone	0.678	0.186	3.564
	Low growth zoning	0.325	0.881	5.367
Jilin	High-speed growth zone	0.698	0.189	3.471
	Low growth zoning	0.286	0.816	5.638
Liaoning	High-speed growth zone	0.765	0.179	3.112
	Low growth zoning	0.238	0.796	4.652

**Table 4:** The zoning transition probability matrix and zoning attributes of the 2005-2020 “liquid_*t*_ − eco_*t*_” system.

liquid_*t*_ − eco_*t*_		Zoning transition probability matrix		Zoning attribute
		High-speed growth zone	Low growth zoning	Average duration
Heilongjiang	High-speed growth zone	0.836	0.539	5.112
	Low growth zoning	0.198	0.463	1.855
Jilin	High-speed growth zone	0.690	0.297	3.015
	Low growth zoning	0.326	0.705	3.365
Liaoning	High-speed growth zone	0.874	0.173	7.961
	Low growth zoning	0.127	0.833	5.993

## Data Availability

This article does not cover data research. No data were used to support this study.
